# Performance of GenoType MTBDR*sl* assay for detection of second-line drugs and ethambutol resistance directly from sputum specimens of MDR-TB patients in Bangladesh

**DOI:** 10.1371/journal.pone.0261329

**Published:** 2021-12-16

**Authors:** S. M. Mazidur Rahman, Rumana Nasrin, Arfatur Rahman, Shahriar Ahmed, Razia Khatun, Mohammad Khaja Mafij Uddin, Md. Mojibur Rahman, Sayera Banu

**Affiliations:** 1 Infectious Diseases Division, icddr,b, Dhaka, Bangladesh; 2 Medicinal Chemistry, Monash Institute of Pharmaceutical Sciences, Monash University, Parkville, Victoria, Australia; 3 Department of Epidemiology, Bangladesh University of Health Sciences, Darus Salam, Mirpur, Dhaka, Bangladesh; INSERM U93: INSERM, FRANCE

## Abstract

**Background:**

Rapid and early detection of drug susceptibility among multidrug-resistant tuberculosis (MDR-TB) patients could guide the timely initiation of effective treatment and reduce transmission of drug-resistant TB. In the current study, we evaluated the diagnostic performance of GenoType MTBDR*sl* (MTBDR*sl*) ver1.0 assay for detection of resistance to ofloxacin (OFL), kanamycin (KAN) and ethambutol (EMB), and additionally the XDR-TB among MDR-TB patients in Bangladesh.

**Methods:**

The MTBDR*sl* assay was performed directly on 218 smear-positive sputum specimens collected from MDR-TB patients and the results were compared with the phenotypic drug susceptibility testing (DST) performed on solid Lowenstein-Jensen (L-J) media. We also analyzed the mutation patterns of *gyrA*, *rrs*, and *embB* genes for detection of resistance to OFL, KAN and EMB, respectively.

**Results:**

The sensitivity and specificity of the MTBDR*sl* compared to phenotypic L-J DST were 81.8% (95% CI, 69.1–90.9) and 98.8% (95% CI, 95.6–99.8), respectively for OFL (PPV: 95.7% & NPV: 94.1%); 65.1% (95% CI, 57.5–72.2) and 86.7% (95% CI, 73.2–94.9), respectively for EMB (PPV: 94.9% & NPV: 39.4%); and 100% for KAN. The diagnostic accuracy of KAN, OFL and EMB were 100, 94.5 and 69.6%, respectively. Moreover, the sensitivity, specificity and diagnostic accuracy of MtBDR*sl* for detection of XDR-TB was 100%. The most frequently observed mutations were at codon D94G (46.8%) of *gyr*A gene, A1401G (83.3%) of *rrs* gene, and M306V (41.5%) of the *emb*B gene.

**Conclusion:**

Considering the excellent performance in this study we suggest that MTBDR*sl* assay can be used as an initial rapid test for detection of KAN and OFL susceptibility, as well as XDR-TB directly from smear-positive sputum specimens of MDR-TB patients in Bangladesh.

## Introduction

The emergence of rifampicin-resistant (RR) or multidrug-resistant (MDR) tuberculosis (TB) has been a significant impediment to the success of global TB control programs. In 2019, an estimated 465,000 incident cases of RR-TB were reported worldwide and 78% of them were MDR-TB. Globally, 3.3% of new and 18% of previously treated TB cases had MDR/RR-TB [1]. Since the end of 2019, the COVID-19 pandemic has severely affected the essential TB services worldwide. WHO analysis of data from 84 countries showed that in the year of 2020 there were about 21% shortfall in the notification of TB cases compared to 2019. The impact of such reduction in TB detection and care may result an estimated half a million of excess death [2]. The absence of early detection of drug-resistant TB may result in treatment failure as well as the development of pre-extensively drug-resistant (pre-XDR) and extensively drug-resistant TB (XDR-TB). XDR-TB is one type of MDR-TB with additional resistance to any of the fluoro-quinolones (FLQ, e.g ofloxacin, moxifloxacin, gatifloxacin, and levofloxacin) and one of the three-second line injectable aminoglycosides (AMG, e.g. kanamycin, amikacin, and capreomycin) [3]. MDR- and XDR-TB account for a significant number of deaths, threaten TB prevention and control programs being an important global health problem. In 2019, a total of 12,350 cases of XDR-TB were reported from 81 countries, and globally 6.2% of MDR-TB patients developed XDR-TB due to the lack of appropriate timely diagnosis and treatment [1]. Bangladesh is also a high TB and MDR-TB burden country with very few cases of TB-HIV co-infection. Despite having a 94% treatment success rate in Bangladesh, 0.7% of new and 11% of previously treated TB cases were either RR- or MDR-TB [1]. Since effective treatment of MDR- and XDR-TB is very costly and they do not respond to the first-line treatment regimens [4]; a rapid, sensitive and specific diagnostic tool is necessary to avoid treatment failure [5].

Conventional phenotypic drug susceptibility testing (DST) on Lowenstein-Jensen (L-J) media is considered as the gold standard method, however, this is slow and requires 4 to 6 weeks to obtain the results [6]. Therefore, rapid, sensitive, and specific methods are required for the detection of *M*. *tuberculosis* as well as determining the drug susceptibility [7, 8]. In 2008, WHO endorsed GenoType® MTBDR*plus* (Hain Lifescience, Nehren, Germany) as a molecular diagnostic test for rapid diagnosis of rifampicin (RIF) and isoniazid (INH) resistance from suspected MDR-TB cases directly from specimens [9]. In May 2016, the WHO recommended the use of molecular probe-based second-line DST assay, the GenoType® MTBDR*sl* ver1.0 (MTBDRT*sl*, Hain Lifescience, Nehren, Germany) to diagnose XDR-TB. This assay can detect the most significant mutations in the *gyrA* gene (responsible for FLQ resistance) and 16S rRNA (*rrs)* gene (responsible for AMG resistance) [10], additionally, it can detect resistance to first-line ethambutol (EMB) drug targeting the *embB* gene. However, the frequency and distribution of mutations vary in contrast to the geographical locations, and so as the performance of the assay [11].

The development of molecular diagnostics could substantially reduce the time of detection for early commencement of appropriate therapy, thus potentially confine drug-resistant-TB transmission. In Bangladesh, a few studies have reported the rapid molecular diagnosis of RR- and MDR-TB by MTBDR*plus* assay and their associated mutation patterns [12–14], however performance evaluation of MTBDR*sl* assay is still lacking. In the current study, we evaluated the performance of MTBDR*sl* assay in contrast to the gold-standard phenotypic DST for the detection of resistance to ofloxacin (OFL), kanamycin (KAN) and EMB, as well as XDR-TB.

## Materials and methods

### Specimens

Sputum specimens were collected from 17 hospitals covering all geographic divisions of Bangladesh, under a nationwide sentinel TB drug resistance surveillance study conducted from 2011 to 2017. By following a systematic random sampling strategy, sputum specimens were collected from newly registered smear-positive pulmonary TB patients. In the current study, only the MDR-TB patients as determined by the phenotypic DST were included for evaluation with MTBDR*sl* assay. The Research Review Committee (RRC) and Ethical Review Committee (ERC) of International Center for Diarrheal Diseases Research, Bangladesh (icddr,b) have approved the study (protocol number: PR-11006). Patients who were already on treatment with anti-TB drugs at the time of diagnosis were excluded from the study. Participants were included in the study only when they agreed to participate and provided written informed consents. For the participans under 18 years of age, consents were obtained from the parents or guardians.

### Specimen processing, culture and drug susceptibility testing

Sputum specimens were decontaminated and processed by following the procedures described previously [15]. Briefly, an equal volume of N-acetyl-L-cysteine (NALC)-NaOH-Na-citrate solution (0.5% NALC, 4% NaOH, and 2.94% Na-citrate) was added to the raw sputum specimen in a 50 ml centrifuge tube and incubated for 15 min at room temperature. The tube was then filled with sterile phosphate-buffered saline (PBS) (pH 6.8) up to 45 ml mark, vortexed well, and centrifuged at 3000g for 15 min. The supernatant was decanted carefully and the resultant sediment was resuspended in 1.0 ml of PBS. Two loops full of processed sputum were then inoculated on two solid L-J slants, incubated at 37°C for up to 8 weeks. The L-J slants were checked once per week and considered culture-positive if colony growth was observed in any of the L-J slants within eight weeks of incubation. If there was no growth after 8 weeks, the specimen was considered as culture-negative. Culture positive *M*. *tuberculosis* isolates were subjected to drug susceptibility testing to OFL (2 μg/μl), KAN (30 μg/μl), and EMB (2 μg/μl) following the standard L-J proportion method as described previously [15]. An isolate was considered resistant to a specific drug when the colony growth of 1% or more was observed in drug-containing media compared to control (drug-free) media.

### GenoType MTBDR*sl* assay

The assay is based on the DNA-strip technology which permits the detection of *M*. *tuberculosis* complex and resistance to FLQ, AMG, and EMB. The assay was performed on decontaminated and concentrated sputum specimens by following the manufacturer’s instructions [16]. Briefly, DNA was extracted from concentrated sputum specimen, amplified by PCR, and the PCR product was hybridized to specific oligonucleotide probes immobilized on the strip. The strip contains six control bands for verification of the test procedures including a conjugate control (CC) band, an amplification control (AC) band, a band specific for *M*. *tuberculosis* complex (TUB), and three locus control bands for drugs (*gyr*A for FLQ, *rrs* for AMG and *emb*B for EMB). The result was considered valid if all the control zones appeared on the strip. An isolate was considered as ‘sensivite’ for a specific drug when all wild-type probes of the respective gene stained positive but no hybridization of any mutant probes within the examined region. Whereas, an isolate was considered as ‘resistant’ when there was the absence of any wild-type probes and/or presence of any mutant probes [16]. In the case of heteroresistant results (strips that showed the presence of bands for both mutation probes and corresponding wild-type probes), we categorized the isolate as “resistant”.

### Quality control

A susceptible strain, H37Rv (ATCC) and our laboratory-defined resistant strain, SB256 were used as quality control for both phenotypic DST and MTBDr*sl* assay. The H37Rv strain was susceptible and SB256 strain was resistant to EMB, OFX, and KAN.

### Statistical analysis

The sensitivity, specificity, positive predictive value (PPV), negative predictive values (NPV), and accuracy of MTBDR*sl* were determined by comparing with phenotypic solid DST method for detection of OFL, KAN and EMB resistance. Agreement between the two methods was assessed using Cohen’s kappa statistic. The kappa value was interpreted as: <0.2, ‘slight’; 0.21–0.4, ‘fair’; 0.41–0.6, ‘moderate’; 0.61–0.8, ‘substantial’; 0.81–0.99, ‘almost perfect’; and 1.0 ‘perfect’ agreement [17].

## Results

### Demographic and clinical characteristics of the participants

A total of 218 MDR-TB cases were included in this study. Among the participants, 63.8% (n = 139) were male and remaining were female (n = 79). The median age of the participants was 30 years with an interquartile range of 22–40 years and more than half (55.5%) of them were between 21–40 years (Table 1). Around 20% of the cases had previous exposure to TB patient in their daily life. Most of the patients (91.7%) had a previous history of TB and anti-TB treatment. The majority (85.8%) of the MDR-TB patients were from the three divisional regions of Chittagong, Rajshahi and Mymensingh (Individual data points are provided in the S1 Dataset).

**Table 1:** Demographic and clinical characteristics of 218 MDR-TB patients.

Variable	Label	Number of patients (n = 218)	Frequency (%)
**Sex**	Male	139	63.8
	Female	79	36.2
**Age (Years)**	≤20	45	20.6
	21–40	121	55.5
	41–60	46	21.1
	>60	6	2.8
**Smoking**	Yes	63	28.9
	No	155	71.1
**Drug User**	Yes	8	3.7
	No	210	96.3
**Dwelling**	Rural	94	43.1
	Urban	124	56.9
**Exposure to TB patients**	Yes	45	20.6
	No	173	79.4
**Previous History of TB**	Yes	200	91.7
	No	18	8.3
**Previous treatment history**	Yes	200	91.7
	No	18	8.3
**Geographic**	Chittagong	89	40.8
	Rajshahi	60	27.5
	Mymensingh	38	17.5
	Dhaka	19	8.7
	Others (Khulna, Sylhet, Barishal)	12	5.5

### Phenotypic drug susceptibility pattern

Phenotypic DST of OFL, KAN, and EMB was performed for all MDR-TB isolates among which 17.9% (39/218) were susceptible to all three drugs (Table 2). Overall, a total of 127 (58.3%) isolates were resistant to any of the three drugs, and only 3 (1.4%) isolates were resistant to all three drugs tested. Total 122 (55.9%) isolates were resistant to only EMB; 3 (1.4%) were resistant to only OFL and 2 (0.9%) were resistant to KAN only. Contrarily, 48 (22%) isolates were simultaneously resistant to both EMB and OFL. There was only one isolate resistant to both KAN and OFL, which means a total of 4 XDR-TB isolates (1.8%) were identified in this analysis (Fig 1A). We determined 53 (24.3%) pre-XDR-TB cases (51 OFL pre-XDR and 2 KAN pre-XDR) in our study. We also found that almost 80% of the MDR-TB patients were resistant to EMB (Table 2).

**Fig 1:** Venn diagram for comparison of the diagnostic performance between the phenotypic DST and MTBDR*sl* assay. A) Susceptibility results of OFL, EMB, and KAN determined by the phenotypic DST and MTBDR*sl* assay for 218 MDR-TB isolates. MTBDR*sl* assay yielded 3 indeterminate results to AMG, of which one had common indeterminate result to EMB also. B) Agreement between MTBDR*sl* assay and phenotypic DST for the detection of OFL, KAN and EMB susceptibility. OFL, ofloxacin; EMB, ethambutol; KAN, kanamycin; FLQ, fluoroquinolone; AMG, aminoglycoside; FLQ^R^, fluoroquinolone resistant; FLQ^S^, fluoro-quinolone sensitivie; EMB^R^, ethambutol resistant; AMG^IND^, aminoglycoside indeterminate; EMB^IND^, ethambutol indeterminate; Phenotypic-R, resistant by phenotypic DST; Phenotypic-S, sensitive by phenotypic DST; MTBDR*sl*-R, resistant by MTBDR*sl* assay; MTBDR*sl*-S, sensitive by MTBDR*sl* assay.

**Table 2:** Phenotypic drug susceptibility patterns of MDR-TB isolates to OFL, KAN and EMB drugs.

Susceptibility pattern	No. of isolates, n (%)
All susceptible	39 (17.9)
All Resistant	3 (1.4)
Only OFL^R^	3 (1.4)
Only EMB^R^	122 (55.9)
Only KAN^R^	2 (0.9)
OFL^R^ + KAN^R^	1 (0.5)
OFL^R^ + EMB^R^	48 (22.0)

OFL^R^, ofloxacin resistant; KAN^R^, kanamycin resistant; EMB^R^, ethambutol resistant.

#### Comparison of MTBDRsl assay with phenotypic DST

Among 218 isolates 47 (21.6%), 6 (2.8%), and 118 (54.1%) isolates were found to be resistant to FLQ, AMG, and EMB, respectively by MTBDR*sl*. Eighty (36.7%) isolates were sensitive to all three drugs. There were total 3 isolates found indeterminate to AMG, of which one had common indeterminate result to EMB also (Fig 1A). Therefore, a total of 218, 215, and 217 isolates had available results for comparison between MTBDR*sl* and phenotypic DST methods for OFL, KAN, and EMB drugs, respectively (Table 3 and Fig 1B).

**Table 3:** Diagnostic performance of MTBDR*sl* assay compared with phenotypic DST method for detection of OFL, KAN, and EMB susceptibility.

GenoType MTBDR*sl*	Phenotypic DST		Sensitivity % (95% CI)	Specificity % (95% CI)	PPV % (95% CI)	NPV % (95% CI)	Accuracy (%) (95% CI)	k-value
	R	S						
OFL (n = 218)			81.8 (69.1–90.9)	98.8 (95.6–99.8)	95.7 (84.9–98.9)	94.1 (90.2–96.6)	94.5 (90.6–97.1)	0.85
R	45	2						
S	10	161						
KAN (n = 215)			100 (54.1–100)	100 (98.3–100)	100	100	100 (98.3–100)	1.0
R	6	0						
S	0	209						
EMB (n = 217)			65.1 (57.5–72.2)	86.7 (73.2–94.9)	94.9 (89.8–97.5)	39.4 (33.9–45.1)	69.6 (63.0–75.6)	0.36
R	112	6						
S	60	39						
XDR-TB (n = 215)			100 (39.8–100)	100 (98.3–100)	100	100	100 (98.3–100)	1.0
R	4	0						
S	0	211						

R, resistant; S, sensitive; CI, confidence Interval; OFL, ofloxacin; KAN, kanamycin; EMB, ethambutol; XDR-TB, extensively drug-resistant tuberculosis.

The sensitivity, specificity, positive predictive value (PPV) and negative predictive value (NPV) of MTBDR*sl* for detecting OFL susceptibility were 81.8% (95% CI, 69.1–90.9), 98.8% (95% CI, 95.6–99.8), 95.7% (95% CI, 84.9–98.9) and 94.1% (95% CI, 90.2–96.6), respectively; and for EMB were 65.1% (95% CI, 57.5–72.2), 86.7% (95% CI, 73.2–94.9), 94.9% (95% CI, 89.8–97.5), and 39.4% (95% CI, 33.9–45.1), respectively. Whereas, the sensitivity, specificity, PPV, and NPV all were 100% for the detection of KAN susceptibility. The 95% CI for sensitivity ranged from 54.1 to100, and for specificity ranged from 98.3–100. The accuracy of the assay for detecting OFL, KAN, and EMB susceptibility was 94.5%, 100%, and 69.6%, respectively. The MTBDR*sl* showed a ‘perfect’ agreement with phenotypic DST for detection of KAN (k value = 1.0), and an ‘almost perfect’ agreement for OFL susceptibility (k value = 0.85), but a ‘fair’ agreement for detection of EMB susceptibility (k value = 0.36) (Table 3). The sensitivity, specificity, PPV, NPV, and accuracy of MTBDR*sl* for detecting XDR-TB was 100% and the agreement between the methods was found “perfect” (k value = 1.0).

### Mutational profiling by MTBDR*sl* assay

MTBDR*sl* detected 47 (21.6%) isolates as FLQ resistant, and among them, the majority of *gyr*A mutations (46.8%, 22/47) were observed by the presence of MUT3C probe which refers to D94G (Table 4). Other mutations at *gyr*A gene were A90V (25.5%), D94A (6.4%), S91P (6.4%), and D94N/D94Y (6.4%), which were detected by the presence of MUT1, MUT3A, MUT2, and MUT3B probes, respectively. However, there were total of 5 (10.6%) isolates that were found resistant by lacking hybridization at wild-type probes (2 isolates for WT2 and 3 isolates for WT3 probes) and no hybridization at mutant probes (Table 4). MTBDR*sl* revealed that only 6 (2.8%) isolates had *rrs* mutations, hence they were resistant to AMG. Among these AMG resistant isolates, 5 (83.3%) of the *rrs* mutations were A1401G (MUT1). For the remaining one, mutation (G1484T) was determined by hybridization at the MUT2 probe. For three isolates, the susceptibility to AMG could not be evaluated due to the absence of locus control, wild and mutant bands at the *rrs* gene, and therefore considered as indeterminate. Of the 118 EMB resistant isolates, the majority of the mutations (41.5%) were determined by the presence of MUT1B (M306V) in *emb*B gene region. Among other mutations, 33 (28.0%) were M306I (MUT1A) and 35 (29.7%) were due to lack of hybridization at WT probes and without any MUT hybridization. Only one EMB resistant isolate showed the presence of both WT probes and MUT1A (M306I) bands. We could not analyze one isolate for EMB susceptibility due to the absence of all bands at *emb*B gene, thus remained indeterminate (S1 Dataset).

**Table 4:** Mutation pattern of *gyr*A, *rrs*, and *emb*B genes obtained by MTBDR*sl* assay using the sputum specimens from MDR-TB patients.

Drugs	Susceptibility	Gene	Resistant associated probes		Mutation detected	No. of isolates (%)
			WT probes	MUT probes		
FLQ	Resistant (n = 47)	*gyrA*	ΔWT2	MUT1	A90V	12 (25.5)
			ΔWT2	MUT2	S91P	3 (6.4)
			ΔWT2	-	Unknown	2 (4.3)
			ΔWT3	MUT3A	D94A	2 (4.3)
			ΔWT3	MUT3B	D94N/D94Y	3 (6.4)
			ΔWT3	MUT3C	D94G	21 (44.6)
			ΔWT3	-	Unknown	3 (6.4)
			WT	MUT3A+MUT3C	D94A+D94G	1 (2.1)
	Sensitive (n = 171)		WT	-	No mutation	171
AMG	Resistant (6)	*rrs*	ΔWT1	MUT1	A1401G	5 (83.3)
			ΔWT2	MUT2	G1484T	1 (16.7)
	Sensitive (n = 209)		WT	-	No mutation	209
EMB	Resistant (n = 118)	*embB*	ΔWT	MUT1A	M306I	33 (28.0)
			ΔWT	MUT1B	M306V	49 (41.5)
			ΔWT	-	M306I	35 (29.7)
			WT	MUT1A	M306I	1 (0.8)
	Sensitive (n = 99)		WT	-	No mutation	99

FLQ, fluoroquinolone; AMG, aminoglycoside; EMB, ethambutol; WT, wild-type visible bands; ΔWT, absence of wild-type bands; MUT, mutation.

## Discussion

For high TB and MDR-TB burden countries like Bangladesh, a rapid and reliable molecular test is crucial for the detection of second-line anti-TB drug susceptibility. In the current study, we have evaluated the diagnostic performance of MTBDR*sl* assay for detection of OFL, KAN, and EMB susceptibility among MDR-TB patients using sputum specimens. The assay demonstrated higher sensitivity and specificity for determination of susceptibility to OFL (sensitivity-81.8% and specificity-98.8%) and KAN (both sensitivity and specificity-100%), but comparatively lower for EMB (sensitivity-65.1% and specificity-86.7%). This finding is in agreement with other previous studies where the sensitivities of MTBDR*sl* ranged from 75.6% to 94.7% for detection of FLQ resistance in different geographical areas like 75.6% in Vietnam [18], 87% in France [19], 93.1% in India [20], and 94.7% in China [21]. The overall sensitivity and specificity for detecting KAN susceptibility in our study were consistent with previous studies that showed 100% sensitivity and specificity [18, 22], but higher than others [19–21, 23–25]. A recent meta-analysis showed a pooled sensitivity and specificity of 86.2% and 98.6% for FLQ; and 87.0% and 99.5% for AMG using MTBDR*sl* assay ver1.0 [26].

Resistance to FLQ is mostly occurred due to the mutations in the *gyrA* gene at codons 94 and 90, and rarely at codons 88 and 91 [27]. As demonstrated in previous studies, mutation detection rate ranged between 57 to 59% for codon 94, and 31 to 35% for codon 90 [28, 29] which is similar to our study found for codon 94 (57.5%) but lower for codon 90 (25.5%). The most common mutations were at D94G in the *gyr*A gene accounting for 46.8% of all mutations, followed by mutations at A90V (25.5%), which were also observed in other related studies [19, 29, 30]. Moreover, we have found some unknown mutations (i.e. lack of hybridization at WT3 probe and no hybridization among mutant probes), which might be located either within 74–113 codon of quinolone resistance determining region (QRDR), as described by the previous study [31] and not covered by the MTBDR*sl* assay or there may be other mechanisms of developing resistance. We did not find any mutation at D94H (MUT3D) of *gyr*A, which is referred to as rare *in silico* mutant [16, 22].

Previous studies demonstrated that the mutation at A1401G of *rrs* gene was the most common and could be attributed to the high level of resistance to KAN and cross-resistance to amikacin (AMK) and capreomycin (CAP) [32, 33]. In our study, we found 83.3% of the *rrs* gene mutations at A1401G (MUT1) followed by mutation at G1484T (16.7%) for AMG resistance. Similar findings were also observed in other related studies in India and South Korea where A1401G was the most frequently occurring mutation for AMG resistance [22, 34]. A recent study in China showed that 92.3% of the *rrs* gene mutation occurred at A1401G, which is much higher compared to our findings [29].

In our analysis, EMB resistance was detected with a sensitivity of 65% and specificity of 87%. Low performance of MTBDR*sl* for detection of EMB resistance was also observed in other previous studies [5, 18, 19, 29, 30], and which could be the reason for excluding the *embB* gene from the MTBDR*sl* ver2.0 assay [35]. The low sensitivity and specificity of MTBDR*sl* ver1.0 for the detection of EMB resistance highlights the necessity of the development of the alternative and improved reliable rapid method. Now, it is an exigent demand to identify the appropriate targets or mechanisms for developing EMB resistance.

For EMB resistance, the majority of the mutations were observed at M306V (41.5%), followed by mutations at M306I (28.0%) and another 29.7% of resistance was due to the absence of wild type probe with no hybridization at any mutant probes. This finding suggests that the significance of mutation in codon 306 is limited and mutation of other codons may be present throughout the *embB* gene which remained unidentified by MTBDR*sl* assay. By DNA sequencing, several mutations of the *embB* gene were previously reported as well with codon 306 [36]. Only one resistant isolate in our study had both WT and MUT1A (M306I) bands. A recent study in China showed the most common mutations at M306V (62.5%), followed by mutations at M306I (37.5%) [29], which concur with our reported data.

In our study, we discovered that approximately 18% and 35% of isolates that were resistant by phenotypic DST for OFL and EMB, respectively were sensitive to the MTBDR*sl* assay. As molecular tests for drug resistance detection are mainly developed based on the more frequent mutations related to resistance, they are unable to target all possible mutations involved in resistance. Therefore, some resistant strains have remained unidentified. Moreover, alteration of the target genes or changes of the amino acid in the target codons might be the cause of false susceptible results as demonstrated by the other studies for FLQ [23, 37] and EMB [23, 38]. Another possible explanation for this kind of discordance could be the presence of a heterogeneous bacterial population. It is known that if the proportion of resistant cells in a specimen is less than 10%, it will be difficult to diagnose the mutant DNA by molecular tests, whereas the phenotypical methods might give resistant results [39]. The existence of heteroresistance among MDR-TB patients is not unusual as this has already been described at higher frequencies for OFL and EMB resistance in Bangladesh [40]. Besides, mutation patterns differ in different geographical regions and settings due to the involvement of different epigenetic or environmental factors. Common mutations are well known for many drugs, but there are silent mutations that never express a drug resistance phenotype. This kind of silent or non-functional mutations affects the performance of the molecular tests.

Finally, false resistant results of MTBDR*sl* assay were also noted for 2 (1.2%) and 6 (13.3%) isolates declared as susceptible to OFL and EMB, respectively by the conventional DST. Of the 2 OFL resistant isolates, one had a mutation at A90V of *gyr*A gene and another one had the absence of WT2 band without staining any mutant band. Of the 6 EMB resistant isolates, two isolates showed mutation at M306I, one at M306V and another 3 isolates had the absence of WT1 without staining any mutant band. The drug-resistant isolates especially the MDR-TB isolates tend to grow slower in the solid medium compared to susceptible isolates as observed in our previous study [15]. In specimens containing mixed isolates, the fast-growing susceptible strain would appear first in the media compared to resistant one, and performing DST using this culture growth would yield ultimately susceptible results. Whereas, DST by MTBDR*sl* directly from the same clinical specimens may provide resistant or heteroresistant results based on the proportion of the strains present in the specimens. False resistance of the isolates with missing wild and mutant bands can be explained by the presence of synonymous mutations that might prevent the binding of both wild and mutant probes as demonstrated in other studies [41].

There were several limitations to our study. MTBDR*sl* ver1.0 was used which was recently been replaced with the MTBDR*sl* ver2.0. The new assay was redesigned on the previous one with the addition of *gyrB* and *eis* genes for improved detection of FLQ and second-line injectable aminoglycosides, respectively, and excluded the EMB drug [35]. In our study, the MTBDR*sl* ver1.0 had a perfect performance for detection of KAN resistance but had 81.7% sensitivity for OFL. A recent study showed that considering *gyrB* gene analysis, sensitivity for FLQ resistance increased from 82.5 to 84.6% [30]. Since most of the mutations for FLQ resistance occur at QRDR of *gyrA* gene and are less frequently found in *gyrB [42], w*e expect that our findings are not so discriminatory with MTBDR*sl* ver2.0 assay. However, future studies are needed to evaluate the performance of MTBDR*sl* ver2.0 in Bangladesh. Moreover, a small number of KAN resistant and XDR-TB cases were analyzed in our study. Another limitation was that we only used smear-positive sputum from MDR-TB patients. Therefore, the performance of the assay in smear-negative pulmonary TB patients can not be determined.

Although the MTBSR*sl* has some limitations, due to its high performance and short turnaround time, the assay can be considered as an initial test in clinical settings for rapid detection of fluoroquinolone and second-line injectable drugs directly from sputum samples of patients with confirmed rifampicin-resistance TB or MDR-TB. Early diagnosis of drug resistance would allow for the early initiation of appropriate therapy and improved health outcomes of the patients.

In conclusion, the current study represents the first evaluation of GenoType MTBDR*sl* ver1.0 assay in Bangladesh for the detection of second-line drugs and EMB resistance among MDR-TB patients. Due to high performance, the assay can be used as an initial rapid test for early detection of XDR-TB, resistance to KAN and FLQ directly from smear-positive sputum specimens of MDR-TB patients.

## Supporting information

S1 Dataset Individual data points. (XLS)

## References

[1] WHO. Global tuberculosis report 2020. Geneva: World Health Organization; 2020. Licence: CC BY-NC-SA 3.0 IGO. 2020.

[2] WHO. Impact of the COVID-19 Pandemic on TB Detection and Mortality in 2020. Available on-line: https://cdn.who.int/media/docs/default-source/hq-tuberculosis/impact-of-the-covid-19-pandemic-on-tb-detection-and-mortality-in-2020.pdf (accessed on 30 March 2021).

[3] JassalM, BishaiWR. Extensively drug-resistant tuberculosis. The Lancet infectious diseases. 2009;9(1):19–30. doi: 10.1016/S1473-3099(08)70260-3 18990610

[4] GandhiNR, NunnP, DhedaK, SchaafHS, ZignolM, Van SoolingenD, et al. Multidrug-resistant and extensively drug-resistant tuberculosis: a threat to global control of tuberculosis. The Lancet. 2010;375(9728):1830–43. doi: 10.1016/S0140-6736(10)60410-2 20488523

[5] ManingiNE, MalingaLA, AntiabongJF, LekalakalaRM, MbelleNM. Comparison of line probe assay to BACTEC MGIT 960 system for susceptibility testing of first and second-line anti-tuberculosis drugs in a referral laboratory in South Africa. BMC Infectious Diseases. 2017;17(1):795. doi: 10.1186/s12879-017-2898-3 29282012PMC5745758

[6] HeifetsL, CangelosiG. Drug susceptibility testing of Mycobacterium tuberculosis: a neglected problem at the turn of the century [State of the Art]. The international journal of tuberculosis and lung disease. 1999;3(7):564–81. 10423219

[7] HillemannD, Rüsch-GerdesS, RichterE. Evaluation of the GenoType MTBDRplus assay for rifampin and isoniazid susceptibility testing of Mycobacterium tuberculosis strains and clinical specimens. Journal of clinical microbiology. 2007;45(8):2635–40. doi: 10.1128/JCM.00521-07 17537937PMC1951233

[8] FalzonD, JaramilloE, SchünemannH, ArentzM, BauerM, BayonaJ, et al. WHO guidelines for the programmatic management of drug-resistant tuberculosis: 2011 update. Eur Respiratory Soc; 2011. doi: 10.1183/09031936.00073611 21828024

[9] WHO. Policy statement. Molecular line probe assays for rapid screening of patients at risk of multidrug resistant tuberculosis (MDR-TB) [homepage on the Internet]. [cited 2008 June 27].

[10] WHO. The use of molecular line probe assays for the detection of resistance to second-line anti-tuberculosis drugs: policy guidance. World Health Organization, 2016 9241516135.

[11] AvalosE, CatanzaroD, CatanzaroA, GaniatsT, BrodineS, AlcarazJ, et al. Frequency and geographic distribution of gyrA and gyrB mutations associated with fluoroquinolone resistance in clinical Mycobacterium tuberculosis isolates: a systematic review. PLoS One. 2015;10(3):e0120470. doi: 10.1371/journal.pone.0120470 ; PubMed Central PMCID: PMC4376704.25816236PMC4376704

[12] AurinTH, MunshiSK, KamalSM, RahmanMM, HossainMS, MarmaT, et al. Molecular approaches for detection of the multi-drug resistant tuberculosis (MDR-TB) in Bangladesh. PloS one. 2014;9(6):e99810. doi: 10.1371/journal.pone.0099810 24932706PMC4059658

[13] RahmanA, SahrinM, AfrinS, EarleyK, AhmedS, RahmanSM, et al. Comparison of Xpert MTB/RIF assay and GenoType MTBDR plus DNA probes for detection of mutations associated with rifampicin resistance in Mycobacterium tuberculosis. PLoS One. 2016;11(4):e0152694. doi: 10.1371/journal.pone.0152694 27054344PMC4824420

[14] UddinMKM, RahmanA, AtherMF, AhmedT, RahmanSMM, AhmedS, et al. Distribution and Frequency of rpoB Mutations Detected by Xpert MTB/RIF Assay Among Beijing and Non-Beijing Rifampicin Resistant Mycobacterium tuberculosis Isolates in Bangladesh. Infection and Drug Resistance. 2020;13:789. doi: 10.2147/IDR.S240408 32210593PMC7073589

[15] BanuS, RahmanSM, KhanMS, FerdousSS, AhmedS, GratzJ, et al. Discordance across several methods for drug susceptibility testing of drug-resistant Mycobacterium tuberculosis isolates in a single laboratory. J Clin Microbiol. 2014;52(1):156–63. doi: 10.1128/JCM.02378-13 ; PubMed Central PMCID: PMC3911413.24172155PMC3911413

[16] LifeScience. H. GenoType MTBDRsl VER 1.0 instructions for use. Document IFU-317A-03. Nehren, Germany: HAIN LifeScience. Document IFU-317A-03. HAIN LifeScience, Nehren, Germany, 2010.

[17] LandisJR, KochGG. The measurement of observer agreement for categorical data. Biometrics. 1977;33(1):159–74. .843571

[18] KietVS, LanNTN, AnDD, DungNH, van Vinh ChauN, ChinhNT, et al. Evaluation of the MTBDRsl test for detection of second-line-drug resistance in Mycobacterium tuberculosis. Journal of clinical microbiology. 2010;48(8):2934–9. doi: 10.1128/JCM.00201-10 20573868PMC2916598

[19] BrossierF, VezirisN, AubryA, JarlierV, SougakoffW. Detection by GenoType MTBDRsl test of complex mechanisms of resistance to second-line drugs and ethambutol in multidrug-resistant Mycobacterium tuberculosis complex isolates. Journal of clinical microbiology. 2010;48(5):1683–9. doi: 10.1128/JCM.01947-09 20335420PMC2863904

[20] ChandakRJ, MalhotraB, BhargavaS, GoelSK, VermaD, TiwariJ. Evaluation of MTBDRsl for detecting resistance in Mycobacterium tuberculosis to second-line drugs. Int J Tuberc Lung Dis. 2019;23(12):1257–62. doi: 10.5588/ijtld.18.0562 .31931908

[21] LuW, FengY, WangJ, ZhuL. Evaluation of MTBDRplus and MTBDRsl in Detecting Drug-Resistant Tuberculosis in a Chinese Population. Dis Markers. 2016;2016:2064765. doi: 10.1155/2016/2064765 ; PubMed Central PMCID: PMC4976146.27524852PMC4976146

[22] AjbaniK, NikamC, KaziM, GrayC, BoehmeC, BalanK, et al. Evaluation of genotype MTBDRsl assay to detect drug resistance associated with fluoroquinolones, aminoglycosides and ethambutol on clinical sediments. PloS one. 2012;7(11):e49433. doi: 10.1371/journal.pone.0049433 23166667PMC3499545

[23] JavedH, BakulaZ, PlenM, HashmiHJ, TahirZ, JamilN, et al. Evaluation of Genotype MTBDRplus and MTBDRsl Assays for Rapid Detection of Drug Resistance in Extensively Drug-Resistant Mycobacterium tuberculosis Isolates in Pakistan. Front Microbiol. 2018;9:2265. doi: 10.3389/fmicb.2018.02265 ; PubMed Central PMCID: PMC6169422.30319577PMC6169422

[24] LacomaA, Garcia-SierraN, PratC, MaldonadoJ, Ruiz-ManzanoJ, HabaL, et al. GenoType MTBDRsl for molecular detection of second-line-drug and ethambutol resistance in Mycobacterium tuberculosis strains and clinical samples. J Clin Microbiol. 2012;50(1):30–6. doi: 10.1128/JCM.05274-11 ; PubMed Central PMCID: PMC3256720.22075597PMC3256720

[25] GaoY, ZhangZ, DengJ, MansjöM, NingZ, LiY, et al. Multi-center evaluation of GenoType MTBDRsl line probe assay for rapid detection of pre-XDR and XDR Mycobacterium tuberculosis in China. Journal of Infection. 2018;77(4):328–34. doi: 10.1016/j.jinf.2018.06.014 29969597

[26] TheronG, PeterJ, RichardsonM, WarrenR, DhedaK, SteingartKR. GenoType® MTBDRsl assay for resistance to second‐line anti‐tuberculosis drugs. Cochrane Database of Systematic Reviews. 2016;(9). doi: 10.1002/14651858.CD010705.pub3 27605387PMC5034505

[27] AubryA, VezirisN, CambauE, Truffot-PernotC, JarlierV, FisherLM. Novel gyrase mutations in quinolone-resistant and-hypersusceptible clinical isolates of Mycobacterium tuberculosis: functional analysis of mutant enzymes. Antimicrobial Agents and Chemotherapy. 2006;50(1):104–12. doi: 10.1128/AAC.50.1.104-112.2006 16377674PMC1346799

[28] LiJ, GaoX, LuoT, WuJ, SunG, LiuQ, et al. Association of gyrA/B mutations and resistance levels to fluoroquinolones in clinical isolates of Mycobacterium tuberculosis. Emerg Microbes Infect. 2014;3(3):e19. doi: 10.1038/emi.2014.21 ; PubMed Central PMCID: PMC3974338.26038513PMC3974338

[29] JianJ, YangX, YangJ, ChenL. Evaluation of the GenoType MTBDRplus and MTBDRsl for the detection of drug-resistant Mycobacterium tuberculosis on isolates from Beijing, China. Infection and Drug Resistance. 2018;11:1627. doi: 10.2147/IDR.S176609 30319279PMC6171507

[30] ZengX, JingW, ZhangY, DuanH, HuangH, ChuN. Performance of the MTBDRsl Line probe assay for rapid detection of resistance to second-line anti-tuberculosis drugs and ethambutol in China. Diagnostic microbiology and infectious disease. 2017;89(2):112–7. doi: 10.1016/j.diagmicrobio.2016.06.011 27345127

[31] TakiffHE, SalazarL, GuerreroC, PhilippW, HuangWM, KreiswirthB, et al. Cloning and nucleotide sequence of Mycobacterium tuberculosis gyrA and gyrB genes and detection of quinolone resistance mutations. Antimicrobial agents and chemotherapy. 1994;38(4):773–80. doi: 10.1128/AAC.38.4.773 8031045PMC284541

[32] GeorghiouSB, MaganaM, GarfeinRS, CatanzaroDG, CatanzaroA, RodwellTC. Evaluation of genetic mutations associated with Mycobacterium tuberculosis resistance to amikacin, kanamycin and capreomycin: a systematic review. PloS one. 2012;7(3):e33275. doi: 10.1371/journal.pone.0033275 22479378PMC3315572

[33] HuY, HoffnerS, WuL, ZhaoQ, JiangW, XuB. Prevalence and genetic characterization of second-line drug-resistant and extensively drug-resistant Mycobacterium tuberculosis in Rural China. Antimicrobial agents and chemotherapy. 2013;57(8):3857–63. doi: 10.1128/AAC.00102-13 23733477PMC3719720

[34] ViaLE, ChoS-N, HwangS, BangH, ParkSK, KangHS, et al. Polymorphisms associated with resistance and cross-resistance to aminoglycosides and capreomycin in Mycobacterium tuberculosis isolates from South Korean patients with drug-resistant tuberculosis. Journal of clinical microbiology. 2010;48(2):402–11. doi: 10.1128/JCM.01476-09 20032248PMC2815586

[35] LifeScience. H. GenoType MTBDRsl VER 2.0 instructions for use. Document IFU-317A-01. Nehren, Germany: HAIN LifeScience. 2015.

[36] HuangW-L, ChiT-L, WuM-H, JouR. Performance assessment of the GenoType MTBDRsl test and DNA sequencing for detection of second-line and ethambutol drug resistance among patients infected with multidrug-resistant Mycobacterium tuberculosis. Journal of clinical microbiology. 2011;49(7):2502–8. doi: 10.1128/JCM.00197-11 21562102PMC3147822

[37] BakulaZ, NapiorkowskaA, KaminskiM, Augustynowicz-KopecE, ZwolskaZ, BieleckiJ, et al. Second-line anti-tuberculosis drug resistance and its genetic determinants in multidrug-resistant Mycobacterium tuberculosis clinical isolates. J Microbiol Immunol Infect. 2016;49(3):439–44. doi: 10.1016/j.jmii.2015.04.003 .26117528

[38] HuangWL, ChiTL, WuMH, JouR. Performance assessment of the GenoType MTBDRsl test and DNA sequencing for detection of second-line and ethambutol drug resistance among patients infected with multidrug-resistant Mycobacterium tuberculosis. J Clin Microbiol. 2011;49(7):2502–8. doi: 10.1128/JCM.00197-11 ; PubMed Central PMCID: PMC3147822.21562102PMC3147822

[39] RichterE, Rüsch-GerdesS, HillemannD. Drug-susceptibility testing in TB: current status and future prospects. Expert Review of Respiratory Medicine. 2009;3(5):497–510. doi: 10.1586/ers.09.45 20477339

[40] OperarioDJ, KoeppelAF, TurnerSD, BaoY, PholwatS, BanuS, et al. Prevalence and extent of heteroresistance by next generation sequencing of multidrug-resistant tuberculosis. PLoS One. 2017;12(5):e0176522. doi: 10.1371/journal.pone.0176522 ; PubMed Central PMCID: PMC5436647.28545050PMC5436647

[41] AjileyeA, AlvarezN, MerkerM, WalkerTM, AkterS, BrownK, et al. Some Synonymous and Nonsynonymous gyrA Mutations in Mycobacterium tuberculosis Lead to Systematic False-Positive Fluoroquinolone Resistance Results with the Hain GenoType MTBDRsl Assays. Antimicrob Agents Chemother. 2017;61(4). doi: 10.1128/AAC.02169-16 ; PubMed Central PMCID: PMC5365657.28137812PMC5365657

[42] OudghiriA, KarimiH, ChetiouiF, ZakhamF, BourkadiJE, ElmessaoudiMD, et al. Molecular characterization of mutations associated with resistance to second-line tuberculosis drug among multidrug-resistant tuberculosis patients from high prevalence tuberculosis city in Morocco. BMC infectious diseases. 2018;18(1):98. doi: 10.1186/s12879-018-3009-9 29486710PMC5830342

